The article "Pairwise Biological Network Alignment Based on Discrete Bat Algorithm" was published in 2021. Journal: Comput Math Methods Med.

# Pairwise Biological Network Alignment Based on Discrete Bat Algorithm

**DOI:** 10.1155/2021/5548993

**Published:** 2021-11-03

**Authors:** Jing Chen, Ying Zhang, Jin-Fang Xia

**Affiliations:** ^1^School of Artificial Intelligence and Computer Science, Jiangnan University, Wuxi, Jiangsu 214122, China; ^2^Jiangsu Provincial Engineering Laboratory of Pattern Recognition and Computing Intelligence, Jiangnan University, Wuxi, Jiangsu 214122, China

## Abstract

The development of high-throughput technology has provided a reliable technical guarantee for an increased amount of available data on biological networks. Network alignment is used to analyze these data to identify conserved functional network modules and understand evolutionary relationships across species. Thus, an efficient computational network aligner is needed for network alignment. In this paper, the classic bat algorithm is discretized and applied to the network alignment. The bat algorithm initializes the population randomly and then searches for the optimal solution iteratively. Based on the bat algorithm, the global pairwise alignment algorithm BatAlign is proposed. In BatAlign, the individual velocity and the position are represented by a discrete code. BatAlign uses a search algorithm based on objective function that uses the number of conserved edges as the objective function. The similarity between the networks is used to initialize the population. The experimental results showed that the algorithm was able to match proteins with high functional consistency and reach a relatively high topological quality.

## 1. Introduction

With the development of high-throughput technology, such as the yeast two-hybrid system [1], an increasing amount of biological data are being modeled into biological networks. According to the different meanings of nodes and edges when the networks are built, the networks can be classified as protein-protein interaction (PPI) networks [2], gene regulatory networks [3], and metabolic networks [4]. Biological systems complete a series of biological processes through PPI, rendering the study of PPI networks of great significance [5]. Network alignment is a more efficient method for analyzing biological networks, in comparison to biological experiments [6], and can be used to discover functional modules among networks [7] and predict the unknown function of proteins [8]. Homologous protein pairs of less-studied biological networks can be discovered by comparison with biological networks that have been more extensively studied, to detect potential functions of unknown proteins [9, 10].

An aspect of the difference of biological network alignment from graph matching is that the goal is the production of biologically meaningful alignment results. Therefore, the sequence similarity, which is an internal property of proteins [11, 12], between network nodes needs to be used in biological alignment. Moreover, the topological structure information of the network, which is an external attribute of proteins, can also be incorporated. The majority of the PPI network alignment algorithms use a combination of sequence similarity and topological similarity [13–15].

Network alignment can be divided into local and global alignment, according to the alignment range [16, 17]. The purpose of local network alignment is to discover similar local subgraphs among networks [18]. MaWISH [19], Graemlin [20], PathBLAST [21], NetworkBLAST [22], and LePrimAlign [23] are examples of algorithms that can be used to solve the local network alignment problem. However, the disadvantage of local network alignment is that one module may be similar to several modules and a protein may be mapped to dissimilar protein nodes [24]. Therefore, the concept of global network alignment has been proposed [25]. Global network alignment is aimed at discovering the overall similar mapping relationship between networks [26]. At present, a high number of global alignment algorithms have been proposed, such as IsoRank [25], GRAAL family algorithms [27–30], NETAL [31], MAGNA [32], MAGNA++ [33], SANA [34], ModuleAlign [35], AligNet [36], and IBNAL [37]. In IsoRank, the similarity of nodes between the networks calculated by the PageRank algorithm is used to guide the greedy algorithm to complete the alignment. The GRAAL family of algorithms includes GRAAL, MI-GRAAL, C-GRAAL, and L-GRAAL, all of which are based on the Graphlet degree similarity. NETAL first constructs an alignment score matrix, and then, a greedy strategy is adopted to update the scores until all nodes in the first network are aligned with nodes in the second network. MAGNA is an objective function-based alignment algorithm that uses a genetic algorithm for searching. MAGNA++ is the optimization of MAGNA that optimizes both structure and sequence similarities and provides a friendly graphical interface. SANA is also objective function-based and uses the simulated annealing search algorithm for alignment. Both the ModuleAlign and AligNet algorithms incorporate the idea of modularity into network alignment. IBNAL develops a clique-based index to measure the topology of the proteins.

Within the framework of objective function-based search algorithms, this paper discretizes the bat algorithm [38] and proposes the BatAlign algorithm. First, the similarity matrix is constructed by the combination of biological similarity and topological similarity information. The sequence similarity adopts BLAST bit-score [39] and evaluates the similarity of the network structure by considering the neighbors of the nodes, to further improve the similarity between networks. The greedy search is then used to generate the initial population, and the pair of nodes with the maximum score is chosen and aligned to each other. Finally, the alignment results are obtained by initial population optimization. By building a coarse similarity score matrix to guide the initialization, BatAlign can shorten the search time to convergence, in comparison to random initialization of the population. Our main contributions are summarized as follows.

1. We propose BatAlign which uses a discrete bat algorithm for network alignment. The main idea of BatAlign is to iteratively update the bat position under the guidance of bat velocity
2. The network topology information and node sequence information are combined to calculate the node similarity. The node similarity guides the construction of the initial population. With the initialization mechanism, BatAlign can obtain a good biological score and relatively high topological score

The related work on network alignment is introduced in the first section. The framework and theory of the BatAlign algorithm are explained in the second section. In the third section, BatAlign is compared with other state-of-the-art algorithms based on synthetic and real networks. The work of this paper and future prospects are presented in Section 4.

## 2. Materials and Methods

### 2.1. Problem Definition

Assume that the two networks to be aligned are *G*_1_(*V*_1_, *E*_1_) and *G*_2_(*V*_2_, *E*_2_), where *V*_1_, *V*_2_ are the node sets of networks *G*_1_, *G*_2_, respectively, and *E*_1_, *E*_2_ are the edge sets of *G*_1_, *G*_2_, respectively. Without loss of generalization, assuming that ∣*V*_1_ | ≤∣*V*_2_∣, the small network *G*_1_ is the source network and the large network *G*_2_ is the target network. Global network alignment finds a mapping relationship *f* : *V*_1_⟶*V*_2_, which aligns the nodes in the small network to the nodes in the large network one by one, to maximize the overall similarity between the networks.

The similarity of the node pairs between networks usually combines the similarity of topology and sequence. In this paper, the topology of the network is considered through the neighbors of a node, and the sequence similarity is combined to generate the similarity matrix between the networks:

(1) $$\begin{array}{c} S=\alpha B+\left(1-\alpha \right)A_{1}BA_{2}^{T},\;\alpha \in \left[0,1\right], \end{array}$$

where *S* represents the similarity matrix between networks, *B* represents the sequence similarity matrix of nodes between networks, and *A*_1_ and *A*_2_ that note the topological structure of the node represent the adjacency matrix of networks *G*_1_ and *G*_2_, respectively.

### 2.2. Bat Algorithm

The bat algorithm [38] is a swarm intelligence optimization algorithm that simulates the echolocation behaviour of bats. The initial population is generated randomly, and then, the optimal solution is iteratively searched. The new solution is generated during searching by adjusting frequency *f* (Equations (3) and (4)); when the rate of pulse emission *r* is smaller than a random number, the local solution is generated around the selected best solution (Equation (5)):

(2) $$\begin{array}{c} f_{i}=f_{\min}+\left(f_{\max}-f_{\min}\right)\;\beta ,\;\beta \in \left[0,1\right], \end{array}$$

(3) $$\begin{array}{c} v_{i}^{t}=v_{i}^{t-1}+\left(x_{i}^{t}-x_{*}\right)f_{i}, \end{array}$$

(4) $$\begin{array}{c} x_{i}^{t}=x_{i}^{t-1}+v_{i}^{t}, \end{array}$$

(5) $$\begin{array}{c} x_{\text{new}}=x_{\text{old}}+\varepsilon A^{t},\;\varepsilon \in \left[-1,1\right]. \end{array}$$

The bats can adjust the loudness (Equation (6)) and the rate of pulse emission (Equation (7)):

(6) $$\begin{array}{c} A_{i}^{t}=\theta A_{i}^{t-1},\;\theta \in \left(0,1\right), \end{array}$$

(7) $$\begin{array}{c} r_{i}^{t}=r_{i}^{t}\left[1-\exp\left(-\gamma t\right)\right],\;\gamma >0. \end{array}$$

### 2.3. Algorithm Overview

#### 2.3.1. Individual and Population Initialization

The BatAlign algorithm applies the discretized bat algorithm to the network alignment, which is reflected in two aspects: position coding and velocity coding.

*Position discretization*: in both networks, the nodes are numbered from one and each node number is unique in its own network. Each individual position in the population represents an alignment of the entire network, the position is a vector *X* with *n*_1_ components, and the entries are members of *G*_2_.

*Velocity discretization*: an individual velocity is represented by a vector *V* with *n*_1_ components, whose entries are 0 or 1. The values 0 or 1 were used to represent the flying velocity of one node in a network, where 0 means keeping the solution of this node, namely, not to fly, and 1 means that the solution of this node can randomly fly.

*Individual initialization*: the position and velocity of each individual need to be initialized. The initial position is an alignment generated by the greedy algorithm under the guidance of the similarity matrix. For example, assuming the similarity matrix of two networks has been obtained by Equation (1), the similarity matrix is shown in Figure 1(c). For each node in the source network, BatAlign identifies the node with the highest similarity; therefore, position *x*_*i*_ is obtained, as shown in Figure 1(d). The method for initializing the velocity is given in Equation (8), and the velocity of the conserved node is 0. For example, assuming the individual position, shown in Figure 2(b), has been obtained, the velocity is obtained as shown in Figure 2(c):

(8) $$\begin{array}{c} v_{k}=\left\{\begin{array}{cc} 0, & \exists \left(u_{k},u_{l}\right)\in E_{1},\exists \left(\emptyset \left(u_{k}\right),\emptyset \left(u_{l}\right)\right)\in E_{2},\\ 1, & \text{otherwise}. \end{array}\right. \end{array}$$

Due to the incompleteness of the similarity between network nodes, it is possible that simple greedy algorithms may not directly align all the nodes. Therefore, unaligned nodes were randomly mapped to generate all the individuals in the population (Figure 3). That is, only the nodes that have similarity are aligned first, while the nodes that do not have similarity are aligned randomly.

#### 2.3.2. Individual and Population Iteration

The individual iteration process is composed of two parts: generating new individuals and updates.

Generating new individuals includes two parts: updating velocity and position. For an individual, the method for updating the velocity is given in

(9) $$\begin{array}{c} v_{ij}^{t}=\left\{\begin{array}{cc} v_{ij}^{t-1}, & \text{if }x_{ij}=x_{*j},\\ {}^{{}^{\circ}}v_{ij}^{t-1}, & \text{otherwise}, \end{array}\right. \end{array}$$

where *v*_*ij*_^*t*^ is the velocity of the *i*th individual on the *j*th dimension during the *t*th iteration, *x*_*ij*_ is the position of the *i*th individual on the *j*th dimension, and *x*_∗*j*_ is the optimal solution on the *j*th dimension. The calculation of °*v*_*ij*_^*t*−1^ is as follows in

(10) $$\begin{array}{c} {}^{{}^{\circ}}v_{ij}^{t-1}=\left\{\begin{array}{cc} {}^{{}^{\circ}}f_{i}, & \text{if }v_{ij}^{t-1}=1,\\ 0, & \text{otherwise}, \end{array}\right. \end{array}$$

where °*f*_*i*_ is calculated as follows in

(11) $$\begin{array}{c} {}^{{}^{\circ}}f_{i}=\left\{\begin{array}{cc} 1, & \text{if }f_{i}>0.5*\left(f_{\max}-f_{\min}\right),\\ 0, & \text{otherwise}, \end{array}\right. \end{array}$$

where *f*_max_ and *f*_min_ represent the maximum and minimum frequency, respectively. In BatAlign, *f*_max_ is set equal to 1 and *f*_min_ equal to 0. The calculation of *f*_*i*_ is Equation (2).

The method to update the position depends on the new velocity. An individual velocity entry of 1 means that this node needs to be remapped and the individual position of this node needs to be changed. Updating the position includes two processes: global search and local search. Each individual position is updated through global search. If the rate of the individual is less than a random number between 0 and 1, BatAlign performs a local search. On the other hand, if the objective function value of the position generated by the local search is larger than the value of the position generated by the global search, then the local search position is accepted. The new position is obtained through global and local search, and if the objective function value of the new position is larger than the old position and the current loudness of the individual is greater than the random number between 0 and 1, BatAlign accepts this new position of the individual.  Figure 4 shows the process of individual iteration.

The global search method is given in Equation (12). The node with a velocity of 0 is reserved, and the remaining nodes are those to be aligned and put into set *U*. The selection operation is represented by *σ*.  Figure 5 shows the global search that generates a new position:

(12) $$\begin{array}{c} x_{ij}^{t}=\left\{\begin{array}{cc} \sigma \left(U\right), & \text{if }v_{ij}^{t}=1,\\ x_{ij}^{t-1}, & \text{otherwise}. \end{array}\right. \end{array}$$

The local search method is given in Equation (13), where the set *C* is composed of nodes with a velocity of 1. An example of local search is shown in Figure 6:

(13) $$\begin{array}{c} x_{ij}^{t}=\left\{\begin{array}{cc} \sigma \left(\text{C}\right), & \text{if }v_{ij}^{t}=1,\\ x_{ij}^{t-1}, & \text{otherwise}. \end{array}\right. \end{array}$$

The update operation is performed when the current loudness of the individual is greater than the random number between 0 and 1 and the value of the objective function of the new position is larger. The objects of the update operation include the velocity, position, rate, and loudness. The objective function used in this study is the number of conserved edges. The more conserved edges, the larger the objective function.

In each iteration, the individual with the highest score is chosen as the optimal solution in the population. When BatAlign runs *T* iterations or the optimal solution remains the same after *N* times, the optimal solution is output as the final alignment.

## 3. Results and Discussion

### 3.1. Experimental Dataset

Synthetic networks were used, retrieved from the NAPAbench2 [40], which was a synthetically constructed network alignment benchmark including three types of networks: Crystal Growth (CG), Duplication Mutation Complementation (DMC), and Duplication with Random Mutation (DMR). The number of nodes and edges of the three networks is shown in Table 1.

The dataset of the real networks was obtained from the BioGRID database [41]. The test species includes the Rattus norvegicus (RN), Schizosaccharomyces pombe (SP), Caenorhabditis elegans (CE), and Mus musculus (MM). The information of the real networks is provided in Table 2.

The similarity scores in the BioGRID datasets were BLAST bit scores computed by the BLAST package on NCBI (https://www.ncbi.nlm.nih.gov/). Gene Ontology terms [42] were used as standard functional annotations, and GO annotations were extracted from NCBI's Entrez Gene database [43].

### 3.2. Evaluation Metrics

The network alignment quality was evaluated in two aspects: topology and biology. The edge conservation under an alignment has been evaluated using three measures so far: Edge Correctness (EC) [27], Induced Conservative Structure (ICS) [44], and Symmetric Substructure Score (*S*^3^) [32]. *S*^3^ has been shown to be superior to EC and ICS, since EC only penalizes alignments from sparse graph regions to dense graph regions. ICS only penalizes alignments from dense graph regions to sparse graph regions; however, *S*^3^ considers both aspects simultaneously. *S*^3^ was used to evaluate the topological similarity of an alignment. The higher the *S*^3^ value is, the more analogous structure the alignment has conserved:

*S* ^3^ was proposed in MAGNA, and it is formulated as

(14) $$\begin{array}{c} S^{3}=\frac{\;|\;f\left(E_{1}\right)\;|\;}{\;|\;E_{1}\;|\;+\left|E_{2}\left(G_{2}\left(f\left(V_{1}\right)\right)\right)\right|-\;|\;f\left(E_{1}\right)\;|\;}, \end{array}$$

where *f* : *V*_1_⟶*V*_2_ represents the alignment and ∣*f*(*E*_1_)∣ is the number of edges from the smaller network *G*_1_ that is conserved by alignment. The formulation of *f*(*E*_1_) is as follows in Equation (15). ∣*E*_2_(*G*_2_(*f*(*V*_1_)))∣ is the number of edges from the induced subnet of *G*_2_ with the aligned node set. The formulation of *f*(*V*_1_) is as follows in Equation (16):

(15) $$\begin{array}{c} f\left(E_{1}\right)=\left\{\left(f\left(u\right),f\left(v\right)\right)\;|\;\left(u,v\right)\in E_{1}:\left(f\left(u\right),f\left(v\right)\right)\in E_{2}\right\}, \end{array}$$

(16) $$\begin{array}{c} f\left(V_{1}\right)=\left\{f\left(u\right)\;|\;u\in V_{1},f\left(u\right)\in V_{2}\right\}. \end{array}$$

The network alignment biological quality was evaluated by two measures, including Gene Ontology consistency (GOC) [45] and Average Functional Similarity (AFS) [46]. The high GOC and AFS values indicate the high functional consistency of the alignment.

GOC is based on the Gene Ontology (GO) consistency of the aligned pairs of proteins. GO terms describe some biological properties of a protein such as Cellular Component (CC), Molecular Function (MF), and Biological Process (BP). Proteins with similar GO terms are supposed to be functionally similar. GOC can be computed as follows in

(17) $$\begin{array}{c} \text{GOC}\left(u,f\left(u\right)\right)=\underset{u\in V_{1}}{\sum }\frac{\left|\text{GO}\left(u\right)\cap \text{GO}\left(f\left(u\right)\right)\right|}{\left|\text{GO}\left(u\right)\cup \text{GO}\left(f\left(u\right)\right)\right|}, \end{array}$$

where GO(*u*) denotes the set of GO terms annotating a protein *u*.

AFS is calculated based on the semantic similarity of the GO terms and depends on the distance between them in the ontology. Semantic similarity measures can be used to calculate the functional similarity in each category of BP, MF, and CC. The semantic similarity is calculated using a graph-based method, Wang. The detailed work of the Wang method is illustrated in [47]. AFS is defined as follows in

(18) $$\begin{array}{c} {\text{AFS}}_{c}=\frac{1}{\left|V_{1}\right|}\times \underset{u\in V_{1}}{\sum }s_{c}\left(u,f\left(u\right)\right), \end{array}$$

where *s*_*c*_ is the semantic similarity of nodes *u* and *f*(*u*), for type *c*(*c* ∈ {BP, MF, CC}), calculated by Wang. GoSemSim [48] was used for semantic similarity calculation.

### 3.3. Experimental Results and Analysis

The number of iterations in BatAlign was set to 1000; the size of the population was set to 40; *N* = 10; that is, when the optimal solution is not updated after 10 times, the current optimal solution was output as the final alignment result. BatAlign makes use of parameter *α* in Equation (1), where *α* determines the relative importance of sequence and topological similarity. Meanwhile, *α* = 1 implies that only sequence information was used. In order to ensure the fairness of the comparison, parameter *α* was set to 0.4 in all the algorithms that use alpha to control the weight of topological similarity and sequence score, and this value was also recommended by ModuleAlign.

To verify the effectiveness of the BatAlign, the algorithm was tested on synthetic and real networks and compared to several state-of-the-art algorithms (i.e., NETAL [31], ModuleAlign [35], L-GRAAL [30], MAGNA [27], and IBNAL [37]). NETAL only adopts topological information to construct the alignment. ModuleAlign is an algorithm based on modularity. L-GRAAL is the representative of the GRAAL family algorithms and integrates Graphlet degree similarity and sequence similarity. MAGNA uses a genetic algorithm, only considers the topological similarity, and is based on the objective function. IBNAL makes use of a novel clique-based index.

The performance of the algorithms is evaluated in Figure 7, based on *S*^3^ on the synthetic networks. In CG networks, the performance of BatAlign was inferior compared to L-GRAAL, NETAL, and ModuleAlign, and *S*^3^ of BatAlign was 1.3-120 times higher than IBNAL and MAGNA. In the DMC networks, the score of BatAlign was 0.1-3.8 times higher than NETAL, MAGNA, and IBNAL. In DMR networks, the performance of BatAlign was inferior to ModuleAlign, L-GRAAL, and NETAL. *S*^3^ of BatAlign was 3.8-4.6 times higher than MAGNA and IBNAL. The results show that the quality of the BatAlign is medium.

The algorithms based on the GOC score on the synthetic networks are compared in Figure 8. BatAlign presented good biological scores in DMC, while its score was slightly lower than ModuleAlign, outperforming the other algorithms. The score of BatAlign was lower than ModuleAlign and L-GRAAL in CG and DMC, while its performance was good compared to the other aligners. The topology of the real network is more complex than that of the synthetic network. Although the performance of BatAlign was not as good as ModuleAlign and L-GRAAL in synthetic networks, BatAlign performed well in real networks. BatAlign can identify functionally consistent proteins, which is helpful to biological research.

Figure 9 shows the results of the different algorithms on the real networks. The BatAlign performance with respect to *S*^3^ was low, while BatAlign outperformed other aligners in terms of GOC; in particular, the alignment between RN and MM achieved an excellent biological score, which may be because these two species were closely related in genetic relationship. NETAL performed best with respect to the *S*^3^ score, but it had a very low GOC score, may be because NETAL is a topological-only method; it can realize high topological quality at the expense of the biological quality. However, GOC carries more importance metrics than *S*^3^ as a metric. In Figure 9, *S*^3^ of ModuleAlign and MAGNA was higher than BatAlign, but they scored low GOC values, and their alignment result may miss node pairs with high functional similarity. The results showed that BatAlign performed much better than IBNAL in terms of *S*^3^ and GOC scores. The GOC of BatAlign was slightly lower than L-GRAAL when aligning RN and CE. However, BatAlign was superior to L-GRAAL when aligning other networks.

AFS provides an alternative way to describe the biological quality of an alignment.  Figure 10 represents the performance of each aligner in terms of AFS. The AFS of BatAlign was 20-50%, 19-54%, and 11-43% higher than NETAL, ModuleAlign, MAGNA, and IBNAL aligners, in terms of BP, MF, and CC, respectively. The performance of L-GRAAL was higher than BatAlign when mapping RN to CE and CE to MM. On the other hand, BatAlign outperformed L-GRAAL, when mapping other networks. Overall, BatAlign has good biological quality compared to other aligners.

On synthetic networks, BatAlign had high GOC scores among selected aligners and competitive *S*^3^ scores. On real networks, BatAlign performed well in terms of the biological score with a relatively high topological score. Thus, BatAlign reached a relatively high topological quality and a superior biological quality. Experiments showed that BatAlign may be a useful tool for predicting the functions of unknown proteins in less studied species through network alignment with species that have been better studied.

## 4. Conclusions and Prospects

The BatAlign based on a discretized bat algorithm for the global alignment of two networks is proposed in this paper. BatAlign discretizes the bat algorithm and uses 0 or 1 to represent the flying velocity. The population of BatAlign is initialized according to the similarity score matrix. A new solution is generated according to a global and a local search, performed according to velocity. The number of conserved edges is used as the objective function. BatAlign overcomes the shortcoming of other search algorithms based on objective functions that initialize the population randomly and can only rely on a larger population and many iterations to find the optimal solution. The results of BatAlign are comparable to other state-of-the-art aligners. Experiments showed that BatAlign is a pairwise biological network global alignment algorithm that performs well in terms of biological quality. Future work will include parallelization of the BatAlign and expansion from two to multiple networks.

## Figures and Tables

**Figure 1:** Initialization of individual position. In this figure, (a, b) are the source network and target network, respectively; (c) is the similarity matrix. Assuming the similarity matrix has been obtained, according to the matrix, the most similar node pair is chosen, and then, a2 is mapped to b3. Nodes are not aligned repeatedly; then, the most similar node pair is a3 and b4; a3 is mapped to b4; in a similar way, a1 is mapped to b1, and a4 is mapped to b5; thus, the individual position can be obtained as shown in (d).

**Figure 2:** Initialization of individual velocity. Assuming the individual position is as shown in (b), according to the position, the edges (a1, a3) and (a2, a3) are conserved; the nodes a1, a2, and a3 are conserved; thus, the velocity of these nodes is 0. Therefore, the individual velocity can be obtained as shown in (c).

**Figure 3:** Initialization of individual position with population size *n*. Assuming the similarity matrix in (a) has been obtained, according to the matrix, the position is obtained as shown in (b); a2 is mapped to b3; a3 is mapped to b4; a1 is mapped to b1; and a4 is mapped to b5. As nodes are not aligned repeatedly, the matrix is obtained as shown in (c). In this case, the similarities of a5 with other nodes are 0; thus, a5 is randomly aligned with b2, b6, b7, or b8; and a6 is also aligned randomly. By mapping unaligned nodes randomly, the positions of individuals with population size *n* are obtained as shown in (d).

**Figure 4:** The individual iteration process.

**Figure 5:** Example of global search. Assuming an individual position with the velocity shown in (b), according to the global search method, the node for which the velocity is 1 is changed through randomly choosing an unaligned node from *U* = {2, 6, 7, 8}; thus, the updated position is obtained as shown in (c).

**Figure 6:** Example of local search. Assuming an individual position with the velocity shown in (b), according to the local search method, the node for which the velocity is 1 is changed through randomly choosing the node for which the velocity equals to 1 from *C* = {4, 6}; thus, the updated position is obtained as shown in (c).

**Figure 7:** *S* ^3^ of the different algorithms on synthetic networks.

**Figure 8:** GOC of the different algorithms on synthetic networks.

**Figure 9:** The performance of the different algorithms on real networks. (a) *S*^3^ and (b) GOC of the different algorithms on real networks.

**Figure 10:** The AFS of the different algorithms on real networks. (a) AFS with respect to BP; (b) MF and (c) CC of the different algorithms on real networks, respectively.

**Table 1:** Information of the synthetic networks. $\bar{k}$ represents the average degree of the network.

Data	Network	Nodes	Edges	$\bar{k}$
CG	A	3000	11987	7.991
	B	4000	15987	7.994

DMC	A	3000	23700	15.8
	B	4000	34206	17.103

DMR	A	3000	30910	20.607
	B	4000	44386	22.193

**Table 2:** Information of the real networks. The species names are mentioned in the first col of the table. The number of nodes and edges are presented in the second and third col, respectively. The fourth col represents the average degree of the network.

Network	Nodes	Edges	$\bar{k}$
RN	2682	4604	3.433
SP	3269	10953	6.701
CE	6058	16463	5.435
MM	7282	21811	5.990

## Data Availability

The data supporting the findings of the article is available at https://github.com/ComplexNetworkJN/BatAlign.
